The article "Adherence to lifelines diet score and risk factors of metabolic syndrome among overweight and obese adults: A cross-sectional study" was retracted in 2024. Reasons: a breach of policy by an author; concerns about the authorship.

# Adherence to lifelines diet score and risk factors of metabolic syndrome among overweight and obese adults: A cross-sectional study

**DOI:** 10.3389/fnut.2022.961468

**Published:** 2022-11-17

**Authors:** Roozbeh Akhavanfar, Ali Hojati, Mohammad Saeed Kahrizi, Mahdieh Abbasalizad Farhangi, Abnoos Mokhtari Ardekani

**Affiliations:** ^1^School of Medicine, Isfahan University of Medical Sciences, Isfahan, Iran; ^2^Department of Community Nutrition, Faculty of Nutrition, Tabriz University of Medical Sciences, Tabriz, Iran; ^3^Alborz University of Medical Sciences, Karaj, Iran; ^4^Tabriz Health Services Management Research Center, Tabriz University of Medical Sciences, Tabriz, Iran; ^5^Endocrinoligy and Metabolism Research Center, Institute of Basic and Clinical Physiology Science and Physiology Research Center, Kerman University of Medical Sciences, Kerman, Iran

**Keywords:** lifeline diet score, metabolic syndivme, obesity, diabetes, cardiovascular diseae

## Abstract

**Background:**

Metabolic syndrome (MetS) is one of the most significant public health issues worldwide, and diet quality is an important controllable environmental factor influencing the incidence of MetS. Numerous dietary scores have been established to assess compliance with dietary recommendations or eating patterns, many of which are not entirely food-based. Hence, Lifelines Diet Score (LLDS) was developed in response to the shortcomings of existing tools. This study aimed to assess any possible links between total food quality and cardiometabolic risk factors among overweight and obese adults.

**Methods:**

This cross-sectional study included 338 overweight and obese individuals [body mass index (BMI) > 25 kg/m^2^] aged 20–50 years in Tabriz, Iran. To collect dietary data, we used a validated semi-quantitative Food Frequency Questionnaire (FFQ) for Iranian population. Enzymatic-colorimetric methods were used to assess serum glucose and lipids, and enzyme-linked immunosorbent assay (ELISA) kits were used to measure insulin levels. In addition, the Homeostasis Model Assessment of Insulin Resistance (HOMA-IR) and Quantitative Insulin Sensitivity Check Index (QUICKI) were calculated.

**Results:**

BMI and hip circumference (HC) were significantly different (*P* < 0.05) amongst LLDS tertiles. Adherence to the highest tertile of LLDS was associated with lower SBP, and the subjects in higher LLDS tertiles significantly had lower systolic blood pressure (SBP) (*P* = 0.04). Triglyceride (TG) levels were also lower in the third tertile of LLDS with a near-significant *P*-value (*P* = 0.05).

**Conclusion:**

According to our results, a higher diet quality score, determined by LLDS, can be associated with a lower risk of MetS. Further experimental and longitudinal studies are needed to better understand this relationship.

The article "Adherence to lifelines diet score and risk factors of metabolic syndrome among overweight and obese adults: A cross-sectional study" was retracted in 2024. Reasons: a breach of policy by an author; concerns about the authorship.

## Introduction

Metabolic syndrome (MetS) is a group of cardiometabolic risk factors primarily characterized by central obesity, insulin resistance, dyslipidemia, hypertension, and hyperglycemia (1). This disorder is linked with increased risk of developing type 2 diabetes (T2D) (2) and cardiovascular disease (CVD) (3, 4). MetS is one of the significant public health issues worldwide because of its rising incidence and poor prognosis, with an upward trend in both industrialized and developing countries (5–7). The global prevalence of MetS in the adult population ranges from 20 to 25% (8); and this rate is 33.7% in Iran (5). Diet quality is given specific consideration as a controllable environmental factor influencing the incidence of MetS (9).

In Iran, there is a significant imbalance in food consumption, with poor nutritional density at all socioeconomic levels (10). According to Iranian dietary habits, it is essential to increase the intake of dairy, fruits, vegetables, grains, poultry, and legumes while decreasing the intake of bread, rice, pasta, red meat, eggs, hydrogenated fats, sugar, and sweets (11). Diet-quality indices allow for assessing a person’s overall diet in relation to specific nutrient consumption, dietary compliance, and risk of chronic disease (12–14).

The Lifelines Diet Score (LLDS), is a food-based diet score developed to examine its capacity to discriminative people with widely different intakes implemented by Vinke et al. (15). LLDS was developed based on the Dutch Dietary Guidelines, and consists of food groups with positive (vegetables, fruits, whole grain products, legumes and nuts, fish, oil and soft margarine, unsweetened dairy products, coffee, and tea), negative (red and processed meat, butter and hard margarine, and sugar-sweetened beverages), neutral, or unknown effects on health (15). As far as the researchers of this study investigated, few studies have investigated the relationship between LLDS adherence and different health conditions. However, the results of the Dutch Lifelines cohort demonstrated that higher adherence to LLDS is associated with a lower all-cause mortality risk in individuals with varying cardiometabolic health levels (16). Also, it has been reported that higher adherence to LLDS is related to decreased odds of breast cancer (17), better sleep quality in obese individuals (18), and reduced T2D incidence (19).

Also, many dietary indexes such as the Healthy Eating Index (HEI), which was developed to reflect the dietary guidelines (20–22), the Mediterranean Diet Score (MDS) (23–25), and the Dietary Approaches to Stop Hypertension (DASH) diet (26) have been established across the world to assess adherence to dietary recommendations and patterns. HEI (27), MDS (28), and DASH diet (29) have been reported to have an inverse association with MetS. Also, the PREDIMED (PREvención con DIeta MEDiterránea) diet score showed an inverse association between adherence to the Mediterranean diet and abdominal or general obesity (30) and CVD (31).

The article "Adherence to lifelines diet score and risk factors of metabolic syndrome among overweight and obese adults: A cross-sectional study" was retracted in 2024. Reasons: a breach of policy by an author; concerns about the authorship.

However, many dietary indexes, including HEI and MDS are not entirely food-based. Thus, in addition to dietary items, these scores also consider the consumption of saturated or unsaturated fatty acids. Furthermore, sugar-sweetened beverages are not included in the MDS, while they have been demonstrated to increase the risk of obesity and diabetes. Accordingly, the LLDS was developed in response to the shortcomings of existing scores, like not being entirely diet-based (15).

Hence, due to limited knowledge on the relationship between LLDS and MetS, further studies are needed to investigate the association between adherence to LLDS and risk factors of MetS. Accordingly, this study aimed to evaluate any possible links between total food quality assessed by LLDS and cardiometabolic risk factors, including lipid profile, glycemic markers, and blood pressure among overweight and obese adults in Tabriz, Iran.

## Materials and methods

### Participants

This cross-sectional study included 338 overweight and obese individuals in Tabriz, Iran. The subjects were selected from two recent projects conducted at Tabriz University of Medical Sciences (32–34). Figure 1 demonstrates the study flowchart. Participants were recruited from the outpatient clinics at the Tabriz University of Medical Sciences by public announcements and distribution of flyers and posters that provided general information about inclusion criteria (age range: 20–50 years; BMI > 25 kg/m^2^) and contact information. The exclusion criteria were pregnancy, breastfeeding, menopausal, recent bariatric surgery, history of CVD, cancer, hepatic or renal disease, diabetes mellitus, and using any drugs affecting weight. All participants signed an informed consent form and the Ethics Committee of Tabriz University of Medical Sciences, Iran approved the study protocol (code: IR.TBZMED.REC.1401.444).

**FIGURE 1:** The study flowchart.

### General characteristics and anthropometric assessments

Using a questionnaire, we collected sociodemographic data, including gender, age, smoking status, educational attainment, marital status, employment, medical history, and family size. Then, socioeconomic status (SES) score was calculated (34). Educational status was measured as ordered categorical variables (illiterate: 0, less than diploma: 1, diploma and associate degree: 2, bachelor’s degree: 3, master’s degree: 4, and higher: 5). In a similar manner, occupation status was also recorded (housewife: 1, employee: 2, student: 3, self-employed: 4 and others: 5 for women; and unemployed: 1, worker, farmer, and rancher: 2, others: 3, employee: 4, and self-employed: 5 for men). Likewise, individuals were classified as having a family size of 3, 4–5, or 6 with scores of 1, 2, and 3, respectively. In addition, they received a score of 1 if they did not own a house and 2 if they owned a house. Finally, each participant received a total SES score between 0 and 15 points.

The article "Adherence to lifelines diet score and risk factors of metabolic syndrome among overweight and obese adults: A cross-sectional study" was retracted in 2024. Reasons: a breach of policy by an author; concerns about the authorship.

Bioelectrical impedance analysis (BIA) was used to determine the body composition (Tanita, BC-418 MA, Tokyo, Japan). Height and weight were determined to the nearest 0.5 cm and 0.1 kg using a wall-mounted stadiometer and a Seca scale (Seca co., Hamburg, Germany), respectively. Physical activity was assessed using a short version of the International Physical Activity Questionnaire (IPAQ) (35). A tape measure was used to determine the waist circumference (WC) to the closest 0.1 cm at the midpoint of the lower costal border and the iliac crest, and the hip circumference (HC) was measured across the broadest section of the buttocks. We also calculated the body mass index (BMI) and waist-hip ratio (WHR). Blood pressure was measured twice in the same arm after at least 15 min of rest using a standard mercury sphygmomanometer (Riester, Diplomat 1002, Jungingen, Germany) and the mean of the two measurements was used for analysis. MetS was defined according to the US National Cholesterol Education Program Adult Treatment Panel III (NCEP-ATP III) criteria (36).

### Dietary assessments tool and its validity-reliability

Dietary data were gathered using a validated semi-quantitative Food Frequency Questionnaire (FFQ) with 168 items for Iranian population (37). The FFQ consisted of a list of items with standard serving sizes Iranians frequently consume. The participants were asked to declare the frequency and quantity of using each food item in a daily, weekly, monthly, or yearly basis. Using standard common portion size available at the manual for Iranian household measures, cooking yields factors and edible portion of foods (38), portion sizes of consumed foods were converted to grams per day (38). For example, one slice of 10*10 cm of Taftoon bread, a traditional Iranian bread, converted to 15 g. The collected data was used to calculate the LLDS. Also, daily dietary intakes were analyzed using NUTRITIONIST IV software (N Squared Computing, California, USA).

The article "Adherence to lifelines diet score and risk factors of metabolic syndrome among overweight and obese adults: A cross-sectional study" was retracted in 2024. Reasons: a breach of policy by an author; concerns about the authorship.

The validity and reliability of the used FFQ were previously assessed (37). Reasonable relative validity was observed based on true estimated validity coefficients, and almost the same correlation coefficient values were observed between men and women for various nutrients. Additionally, to determine the 1-year reliability of the FFQ, the intra-class correlation was calculated. Intra-class correlation coefficients between the two FFQs, administered at a 1-year interval, ranged from 0.41 (monounsaturated fat) to 0.79 (protein) in men and from 0.39 (monounsaturated fat) to 0.74 (saturated fat) in women. In two age groups, ≤ 35 and > 35 years, the mean adjusted intra-class correlation coefficients between the two FFQ were 0.48 and 0.65, respectively (37). For validity assessment, also, the ranges of questionnaire validity coefficients, with the sample correlation between the questionnaires and biochemical marker as the lower limit and the estimate obtained by the method of triads as the upper limit, were 0.21–0.56 (protein), 0.37–0.61 (K), 0.38–0.50 (b-carotene), 0.31–0.95 (cholesterol), 0.21–0.55 (retinol), and 0.28–0.38 (a-tocopherol) (37).

Additionally, this FFQ enables accurate ranking of people according to their food group consumption levels and appears to be an acceptable tool for evaluating food group intake based on its reasonable relative validity and reproducibility correlations. The food items on the FFQ were categorized based on their nutrient contents. The food groups were determined as follows: (1) whole grains, (2) refined grains, (3) potatoes, (4) dairy products, (5) vegetables, (6) fruits, (7) legumes, (8) meats, (9) nuts and seeds, (10) solid fat, (11) liquid oil, (12) tea and coffee, (13) salty snacks, (14) simple sugars, (15) honey and jams, (16) soft drinks, and (17) desserts and snacks (39).

Dietary salt consumption was evaluated by asking about frequency of adding salt or salty sauce to food during preparation/cooking, or before or while eating and/or frequency of consuming high-salt processed foods.

### Calculation of the lifelines diet score

Based on Vinke et al. (15) and the LLDS standards, foods were grouped into positive, negative, neutral, or unknown categories according to their impact on health. Vegetables, fruits, whole grain products, legumes and nuts, fish, oils and soft kinds of margarine, unsweetened dairy, coffee, and tea constituted positive groups. On the other hand, negative food groups included red and processed meat, butter and hard margarine, and sugar-sweetened drinks. There were also nine unknown categories, including potatoes, refined grain products, unprocessed white meat, cheese, ready and savory foods, sugary products, soups, sweetened dairy, and artificially sweetened products, as well as a neutral group of eggs. The LLDS was constructed using the positive and negative food groups. The dietary intake of food groups was stated in grams per 1,000 kilocalories rather than grams per day to consider the differences between participants’ caloric intake, and the findings were divided into quintiles of 1–5, with 1 indicating the lowest intake and 5 indicating the highest intake. The overall LLDS score ranged from 12 to 60 based on the 12 element scores.

The article "Adherence to lifelines diet score and risk factors of metabolic syndrome among overweight and obese adults: A cross-sectional study" was retracted in 2024. Reasons: a breach of policy by an author; concerns about the authorship.

### Biochemical assessment

For biochemical assessment, 10 ml of fasting venous blood was collected from all participants. Serum and plasma samples were separated by centrifugation at 4,500 rpm for 10 min at 4^°^C. Until analysis, aliquots were frozen at −70^°^C. A commercial kit was used to determine total serum cholesterol (TC), triglyceride (TG), high-density lipoprotein cholesterol (HDL-C), and fasting blood glucose (FBG) (Pars Azmoon, Tehran, Iran). Additionally, to determine the amount of low-density lipoprotein cholesterol (LDL-C), the Friedewald equation was applied (40). Blood insulin levels were evaluated by enzyme-linked immunosorbent assay (ELISA) kits (Bioassay Technology Laboratory, Shanghai Korean Biotech, Shanghai City, China). The Homeostasis Model Assessment of Insulin Resistance (HOMA-IR) was determined by fasting insulin (IU/ml)/22.5 fasting glucose (mmol/l), and the Quantitative Insulin Sensitivity Check Index (QUICKI) was calculated using the following formula: 1/[log fasting insulin (U/mL) + log glucose (mmol/L).

### Statistical analysis

The data were analyzed using SPSS version 26.0 at a significance level of 0.05. The frequency (percentage) was reported for categorical data, and mean and standard deviation (SD) were provided for continuous variables. A general linear model was used to assess the changes in variables among different tertiles of LLDS. Additionally, the association between the LLDS tertiles and biochemical variables was assessed using multinomial logistic regression to estimate odds ratios (ORs) and 95% confidence intervals (CIs) for the presence of cardiometabolic risk factors across the LLDS tertiles in two multivariable-adjusted models.

Because no study has investigated the relationship between LLDS and MetS, we calculated the sample size based on the study of Kesse-Guyot et al. (41), which investigated the association of MDS and the risk of MetS (OR = 0.44, 95% CI = 0.29–0.67). According to this study, the odds ratio of MetS was considered the main basis for calculating the sample size. The sample size of the current study was calculated using the following formula for the absence group (the group with the lowest diet quality score): n_*a*_ = [Z_α__/2_^2^/log^2^(1-RP)] * [1/X + 1/Y], where, X = 1/ρ_*p*_(1-ρ_*p*_)k, and Y = 1/ρ_*a*_(1-ρ_*a*_) with considering a confidence interval of 95% (α = 0.05), and relative precision (RP) of 48%. ρ_*p*_ is the prevalence of the outcome in the presence group (the group with the highest diet quality score), ρ_*a*_ is the prevalence of the outcome in the absence group, and k is the ratio of presences to absences being sampled (n_*p*_/n_*a*_). The prevalence of MetS in the Iranian adult population is 33.7%, and the ratio of presences to absences being sampled is one. Accordingly, the calculated sample size was estimated as 303 individuals. Considering the drop-out rate of 11%, a total of 338 samples were entered into the study.

The article "Adherence to lifelines diet score and risk factors of metabolic syndrome among overweight and obese adults: A cross-sectional study" was retracted in 2024. Reasons: a breach of policy by an author; concerns about the authorship.

## Results

The current study included 338 participants (aged 40.78 ± 9.23 years) with a mean BMI of 32.63 ± 4.81 kg/m^2^. Table 1 outlines the participants’ characteristics by LLDS tertiles. While BMI and HC were significantly different (*P* < 0.05) amongst LLDS tertiles, weight, height, WC, WHR, FM, FFM, BMR, and physical activity levels were not significantly different (*P* > 0.05). However, no significant differences were found after multivariable adjustment. The subjects in higher LLDS tertiles significantly had lower systolic blood pressure (SBP) (*P* = 0.04), and TG levels were lower in the third tertile of LLDS, with a near-significant *P*-value (*P* = 0.05). However, TG levels in the second tertile were higher than in the first tertile. Conversely, no significant differences (*P* > 0.05) were seen between LLDS tertiles and diastolic blood pressure (DBP), TC, HDL-C, LDL-C, glucose, insulin, HOMA-IR, and QUICKI. However, after multivariable adjustment, no significant differences were found for cardiometabolic risk factors across tertiles of LLDS (Table 2).

**TABLE 1:** Demographic and anthropometric characteristics of participants across different tertiles of LLDS.

Variables	Tertiles of LLDS, mean (*SD*)			*P*-value	*P*-value*
	1st tertile (*n* = 112)	2nd tertile (*n* = 114)	3rd tertile (*n* = 112)		
Age (year)	38.54 (9.72)	40.48 (8.66)	42.58 (9.11)	**0.022**	**–**
Weight (kg)	91.09 (13.15)	93.47 (15.06)	90.81 (14.49)	0.512	0.367
Height (cm)	169.82 (9.63)	168.53 (9.46)	165.37 (10.35)	**0.008**	0.767
BMI (kg/m^2^)	31.67 (4.48)	32.93 (50.10)	33.11 (4.62)	0.410	0.487
Sex [male *n* (%)]	72 (64.28)	66 (57.89)	56 (50.00)	0.125	–
SES score	9.98 (2.51)	10.07 (2.44)	9.80 (2.64)	0.832	–
WC (cm)	105.76 (8.55)	107.66 (10.12)	106.00 (9.60)	0.526	0.333
HC (cm)	112.81 (10.00)	116.03 (9.77)	114.89 (7.55)	0.282	0.142
WHR	0.94 (0.08)	0.94 (0.08)	0.92 (0.07)	0.075	0.188
FM (kg)	31.83 (7.2)	34.93 (10.79)	33.69 (7.41)	0.780	0.251
FFM (kg)	63.50 (12.34)	63.29 (12.43)	59.58 (12.05)	0.155	0.912
BMR (kcal)	1973.53 (519.65)	1926.99 (350.59)	1812.90 (333.22)	0.120	0.721
PA (MET. min/week)	1952.48 (3254.71)	2149.90 (3182.71)	2413.23 (3270.66)	0.743	–

BMI, body mass index; WC, waist circumference; HC, hip circumference; WHR, waist to hip ratio; FM, fat mass; FFM, fat free mass; BMR, basal metabolic rate; PA, physical activity. All data are expressed as mean (±*SD*). *P*-values derived from one-way ANOVA. *Anthropometric variables were adjusted for demographic characteristics including age, sex, socioeconomic status, and physical activity. The bold values represent statistically significance.

The article "Adherence to lifelines diet score and risk factors of metabolic syndrome among overweight and obese adults: A cross-sectional study" was retracted in 2024. Reasons: a breach of policy by an author; concerns about the authorship.

**TABLE 2:** Cardiometabolic components of participants across different tertiles of LLDS.

Variables	Tertiles of LLDS, mean (*SD*)			*P*-value	*P*-value*
	1st tertile (*n* = 112)	2nd tertile (*n* = 114)	3rd tertile (*n* = 112)		
SBP (mmHg)	124.26 (16.07)	123.06 (14.64)	120.77 (18.41)	**0.040**	0.870
DBP (mmHg)	81.15 (10.53)	81.61 (11.28)	81.99 (11.71)	0.934	0.678
TC (mg/dL)	192.53 (32.67)	192.38 (37.53)	190.23 (39.23)	0.401	0.243
TG (mg/dL)	147.83 (82.39)	162.05 (101.67)	135.28 (86.99)	**0.050**	0.349
HDL-C (mg/dL)	43.95 (8.44)	42.50 (9.87)	44.77 (9.75)	0.175	0.489
LDL-C (mg/dL)	123.41 (30.80)	122.99 (30.14)	124.72 (35.94)	0.958	0.401
Glucose (mg/dL)	91.88 (16.46)	93.29 (23.66)	92.78 (13.78)	0.890	0.560
Insulin (μ IU/mL)	13.87 (8.23)	17.76 (17.12)	15.33 (10.40)	0.165	0.582
HOMA-IR	3.21 (2.10)	4.20 (4.00)	3.50 (2.65)	0.114	0.265
QUICKI	0.34 (0.04)	0.32 (0.03)	0.33 (0.04)	0.083	0.713

SBP, systolic blood pressure; DBP, diastolic blood pressure; TC, total cholesterol; TG, triglyceride; HDL, high density lipoprotein; LDL, low density lipoprotein; HOMA-IR, homeostatic model assessment for insulin resistance; QUICKI, quantitative insulin-sensitivity check index. All data are expressed as mean (±*SD*). *P*-values derived from one-way ANOVA. *All variables were adjusted for demographic characteristics including age, sex, socioeconomic status, and physical activity. The bold values represent statistically significance.

The average dietary intake of subjects in different LLDS tertiles is represented in Table 3. Total fat (*P* = 0.013), cholesterol (*P* = 0.010), sodium (*P* = 0.004), iron (*P* = 0.020), selenium (*P* = 0.002), vitamin B1 (*P* = 0.005), vitamin B3 (*P* = 0.005), vitamin B9 (*P* = 0.024), and monounsaturated fatty acids (*P* = 0.030) intakes were significantly lower among different tertiles, and vitamin D intake (*P* = 0.002) was significantly higher across LLDS tertiles. Table 4 shows the dietary intake of 12 LLDS components (grams/1,000 kcal) among participants in different LLDS tertiles. As can be seen, the consumption rate of whole grains, fruits, vegetables, fish, legumes, and nuts, unsweetened dairy, and tea was significantly higher in greater LLDS tertiles. In contrast, the consumption rate of red and processed meat consumption, butter and hard margarines, and sugar-sweetened beverages was lower in greater LLDS tertiles. Table 5 demonstrates the crude and multivariable adjusted odds ratios (ORs) and 95% confidence interval (CI) for risk factors of MetS across different tertiles of LLDS. Participants in the highest tertile of LLDS had lower odds of SBP in the adjusted model I [OR: 0.983 (0.965–1.001; *P* < 0.05)]. No other significant association was found in crude and multivariable-adjusted models.

The article "Adherence to lifelines diet score and risk factors of metabolic syndrome among overweight and obese adults: A cross-sectional study" was retracted in 2024. Reasons: a breach of policy by an author; concerns about the authorship.

**TABLE 3:** Dietary intakes of participants across different tertiles of LLDS.

Dietary components	Tertiles of LLDS, mean *(SD)*			*P*-value	Dietary components	Tertiles of LLDS, mean *(SD)*			*P*-value
	1st tertile (*n* = 112)	2nd tertile (*n* = 114)	3rd tertile (*n* = 112)			1st tertile (*n* = 112)	2nd tertile (*n* = 114)	3rd tertile (*n* = 112)	
Protein (g/day)	101.21 (45.20)	103.10 (33.75)	93.52 (33.89)	0.127	Manganese (mg/day)	8.43 (4.07)	9.28 (3.81)	8.88 (3.60)	0.258
Fat (g/day)	109.02 (53.63)	103.19 (45.83)	89.45 (40.99)	**0.013**	Selenium (mg/day)	159.38 (73.22)	160.12 (59.78)	133.95 (50.87)	**0.002**
Cho (g/day)	465.84 (194.43)	467.49 (167.77)	416.07 (146.27)	**0.045**	Fluorine (mg/day)	3064.72 (3715.35)	3364.10 (2537.06)	3958.43 (3117.32)	0.122
Total Fiber (g/day)	69.95 (42.54)	68.59 (37.59)	58.73 (35.79)	0.079	Chromium (mg/day)	0.14 (0.11)	0.17 (0.13)	0.15 (0.099)	0.099
SFA (g/day)	31.08 (14.65)	30.31 (15.76)	26.45 (13.66)	0.065	Copper (mg/day)	2.53 (1.46**)**	2.58 (1.10**)**	2.28 (0.90**)**	0.109
MUFA (g/day)	35.50 (18.01)	34.50 (16.77)	29.63 (14.85)	**0.030**	VitaminB1 (mg/day)	2.77 (1.18)	2.73 (0.10)	2.33 (1.01)	**0.005**
PUFA (g/day)	24.98 (15.74)	22.80 (11.73)	20.36 (12.88)	0.060	VitaminB2 (mg/day)	2.57 (1.19)	2.62 (0.96)	2.47 (1.02)	0.518
Cholesterol (mg/day)	328.03 (285.23)	311.55 (178.14)	246.67 (115.22)	**0.010**	VitaminB3 (mg/day)	30.77 (12.52)	30.82 (10.51)	26.45 (10.07)	**0.005**
Trans fatty acids (g/day)	0.0020 (0.0068)	0.0013 (0.0056)	0.0009 (0.0054)	0.494	Vitamin A (RAE/day)	892.80 (852.12)	914.20 (707.16)	890.33 (452.89)	0.955
Sodium (mg/day)	4961.88 (2191.38)	4935.22 (2341.98)	4063.16 (1984.11)	**0.004**	Vitamin D (μ g/day)	1.67 (1.34)	1.98 (1.46)	2.44 (1.63)	**0.002**
Iron (mg/day)	24.38 (10.58)	25.09 (12.14)	21.30 (7.96)	**0.020**	Vitamin K (μ g/day)	212.94 (213.29)	259.34 (239.35)	277.36 (274.31)	0.184
Magnesium (mg/day)	514.05 (298.45)	562.70 (216.19)	539.72 (181.77)	0.292	Vitamin E (mg/day)	15.59 (7.44)	16.92 (8.57)	15.72 (8.64)	0.380
Zinc (mg/day)	15.02 (9.34)	15.33 (6.20)	13.80 (5.07)	0.214	VitaminB6 (mg/day)	2.20 (0.92)	2.43 (0.95)	2.30 (0.83)	0.177
Phosphorus (mg/day)	1725.24 (746.78)	1857.11 (607.86)	1795.69 (664.38)	0.332	VitaminB9 (μ g/day)	746.39 (312.85)	738.26 (290.00)	674.63 (273.24)	**0.024**
Calcium (mg/day)	1219.46 (591.38)	1318.91 (510.67)	1307.93 (629.79)	0.404	VitaminB12 (μ g/day)	6.21 (8.36)	5.45 (5.83)	4.41 (2.78)	0.119
Potassium (mg/day)	4390.73 (2262.02)	4783.24 (2065.65)	4993.18 (1788.65)	0.131	Vitamin C (mg/day)	215.47 (163.51)	241.83 (197.52)	257.78 (160.53)	0.274

SFA, saturated fatty acids; MUFA, mono-unsaturated fatty acids; PUFA, poly-unsaturated fatty acids. All data are expressed as mean (±*SD*). *P*-values derived from one-way ANOVA. The bold values represent statistically significance.

The article "Adherence to lifelines diet score and risk factors of metabolic syndrome among overweight and obese adults: A cross-sectional study" was retracted in 2024. Reasons: a breach of policy by an author; concerns about the authorship.

**TABLE 4:** Consumption rates of 12 Lifelines Diet Score (LLDS) components (grams/1,000 kcal).

	Tertiles of LLDS, mean (SD)				
	1st tertile (*n* = 112)	2nd tertile (*n* = 114)	3rd tertile (*n* = 112)	*P-*value	*P-*value*
LLDS score	29.25 (2.89)	35.51 (1.74)	42.18 (2.99)	** < 0.001**	** < 0.001**
**Positive components**					
Whole grains	36.02 (25.17)	51.10 (37.80)	57.08 (36.23)	** < 0.001**	0.085
Fruits	178.67 (122.34)	214.68 (164.61)	286.01 (200.61)	** < 0.001**	**0.013**
Vegetables	91.07 (45.84)	118.57 (64.94)	163.11 (78.26)	** < 0.001**	** < 0.001**
Fish	2.21 (3.21)	3.34 (4.25)	5.28 (6.05)	** < 0.001**	**0.010**
Legumes and nuts	17.40 (14.28)	23.33 (21.71)	30.61 (18.78)	** < 0.001**	**0.006**
Oils and soft margarines	8.56 (7.52)	9.54 (**??**)	9.27 (8.05)	0.450	0.680
Unsweetened dairy	76.97 (60.62)	100.80 (63.11)	140.46 (75.39)	** < 0.001**	** < 0.001**
Coffee	3.62 (10.18)	7.57 (20.32)	10.02 (16.93)	0.078	0.327
Tea	286.62 (340.06)	302.32 (271.52)	408.75 (311.84)	**0.006**	**0.011**
**Negative components**					
Red and processed meat	16.26 (16.04)	10.66 (8.38)	7.56 (5.64)	** < 0.001**	**0.002**
Butter, hard margarines	1.78 (2.12)	1.26 (1.95)	0.76 (1.20)	**0.005**	**0.024**
Sugar-sweetened beverages	26.39 (33.58)	13.16 (23.57)	6.61 (14.22)	** < 0.001**	** < 0.001**

All data are expressed as mean (±*SD*). *P*-values derived from one-way ANOVA. *All variables were adjusted for demographic characteristics including age, sex, socioeconomic status, and physical activity. The bold values represent statistically significance.

**TABLE 5:** Crude and multivariable adjusted ORs and 95% CIs for cardiometabolic risk factors across different tertiles of LLDS.

Variables	Tertiles of LLDS								
	Crude ORs (95% CI)			Model I^a^ ORs (95% CI)			Model II^b^ ORs (95% CI)		
	1st (*n* = 112)	2nd (*n* = 114)	3rd (*n* = 112)	1st (*n* = 112)	2nd (*n* = 114)	3rd (*n* = 112)	1st (*n* = 112)	2nd (*n* = 114)	3rd (*n* = 112)
SBP (mmHg)	1	0.997 (0.981–1.013)	0.988 (0.972–1.005)	1	0.992 (0.974–1.010)	0.983 (0.965–1.001)*	1	0.997 (0.970–1.025)	0.999 (0.971–1.029)
DBP (mmHg)	1	0.993 (0.972–1.015)	1.000 (0.977–1.024)	1	0.987 (0.964–1.011)	0.994 (0.970–1.018)	1	0.986 (0.953–1.020)	1.008 (0.974–1.044)
FBG (mg/dl)	1	1.006 (0.992–1.020)	1.003 (0.988–1.019)	1	1.004 (0.990–1.018)	0.998 (0.983–1.014)	1	1.008 (0.991–1.025)	0.995 (0.972–1.018)
TC (mg/dL)	1	1.002 (0.995–1.009)	0.999 (0.992–1.007)	1	1.001 (0.992–1.008)	0.999 (0.992–1.006)	1	1.001 (0.990–1.012)	0.995 (0.984–1.007)
LDL–C (mg/dL)	1	1.001 (0.993–1.009)	1.002 (0.993–1.010)	1	1.000 (0.992–1.008)	1.001 (0.993–1.010)	1	1.002 (0.991–1.014)	0.997 (0.985–1.010)
HDL–C (mg/dL)	1	0.980 (0.953–1.007)	1.009 (0.981–1.037)	1	0.976 (0.948–1.006)	0.995 (0.967–1.024)	1	0.977 (0.937–1.019)	0.982 (0.941–1.025)
TG (mg/dL)	1	1.002 (0.999–1.004)	0.998 (0.994–1.001)	1	1.001 (0.998–1.004)	0.999 (0.996–1.003)	1	1.001 (0.995–1.007)	0.998 (0.991–1.005)
Insulin (μIU/mL)	1	1.026 (0.998–1.055)	1.010 (0.979–1.043)	1	1.026 (0.998–1.055)	0.999 (0.968–1.032)	1	1.021 (0.982–1.062)	0.984 (0.943–1.027)

*P < 0.05; ^*a*^Model I, adjusted for age, sex, and BMI; ^*b*^Model II, additionally adjusted for socioeconomic status, and energy intake. SBP, systolic blood pressure; DBP, diastolic blood pressure; FBG, fasting blood glucose; TC, total cholesterol; LDL-C, low density lipoprotein cholesterol; HDL-C, high density lipoprotein cholesterol; TG, triglyceride. The bold values represent statistically significance.

The article "Adherence to lifelines diet score and risk factors of metabolic syndrome among overweight and obese adults: A cross-sectional study" was retracted in 2024. Reasons: a breach of policy by an author; concerns about the authorship.

## Discussion

This cross-sectional study assessed any possible links between adherence to LLDS and cardiometabolic components among Iranian overweight and obese adults. Lower cardiometabolic risk factors could be linked to better adherence to the LLDS, which implies a healthy eating pattern. It is widely recognized that examining the entire diet rather than particular meals or nutrients can provide a more accurate picture of overall diet quality and aid in predicting the link between diet quality and health risks (42–44). It should also be noted that LLDS score is a diet-based index for measuring diet quality.

As the primary finding of this study, a better diet quality score, as determined by higher LLDS with a rise in the consumption of positive food groups and a reduction in the consumption of negative food groups, led to a significantly lower SBP. Likewise, Drewnowski et al. found that a high-quality diet, measured by the HEI, could decrease SBP and DBP in males (45). Consistent with our findings, Tzima et al. evaluated diet quality using the MDS and reported that a high-diet quality led to lower SBP and DBP across different tertiles (46). Additionally, Nicklas et al. demonstrated that persons with the highest diet quality had a lower risk of having hypertension (12). Also, Harrington et al. demonstrated a significant converse association between DASH score and SBP in standardized clinical records (47).

The article "Adherence to lifelines diet score and risk factors of metabolic syndrome among overweight and obese adults: A cross-sectional study" was retracted in 2024. Reasons: a breach of policy by an author; concerns about the authorship.

In this study, dietary intake of sodium was estimated using the sodium content of foods and the amount of table salt consumed. Reduced sodium intake across different tertiles of LLDS might be a probable underlying mechanism between LLDS and lower SBP. As Grillo et al. showed in their review study, numerous studies have established a clear relation between sodium consumption and blood pressure levels (48). The relationship between high sodium consumption and high blood pressure can be explained by various mechanisms, including increased reuptake and retention of sodium in the kidney tubules and activation of the brain renin-angiotensin-aldosterone system. This mechanism is thought to raise blood pressure by increasing angiotensin II and aldosterone levels in the blood while also increasing oxidative stress and activation of the sympathetic nervous system (49). Additionally, according to the “vasodysfunction theory,” excessive sodium intake can lead to defective systemic vascular resistance, which results in a rise in blood pressure (50). Along with blood pressure, a systematic review and meta-analysis of randomized controlled trials found that dietary sodium limitation can decrease arterial stiffness (51). Other probable processes include water retention, a rise in systemic peripheral resistance, endothelial dysfunction, and alterations in sympathetic activity and cardiovascular system autonomic neural control, which all contribute to the relationship between excessive sodium intake and the risk of hypertension (52). Also, as Roberts et al. discussed, eating fruits and vegetables may help decrease blood pressure, defend against lipid peroxidation, and enhance antioxidant capacity, as indicated by enhanced plasma carotenoids and serum oxygen radical-absorbing ability (53) (Figure 2).

**FIGURE 2:** High dietary sodium intake can induce high blood pressure through the renin angiotensin system, which leads the hypothalamus to stimulate thirst and increase water intake. Also, it stimulates anti-diuretic hormone (ADH) secretion from the pituitary gland (77), which increases the aquaporin channels in the collecting duct and distal convoluted tubule (78). A high sodium intake activates extracellular matrix metalloproteinases MMP2 and MMP9, stimulating TGFß-1, inducing thinning and breakage of elastin fibers, and decreasing the elastin and collagen ratio. Also, TGFß-1 inhibits collagenase production and develops a fibrogenic effect on the extracellular matrix in the arterial wall, altering its mechanical properties and causing arterial stiffness (48). Asymmetrical dimethylarginine (ADMA) is a major endogenous inhibitor of NO bioavailability through its capacity to inhibit NO synthase and also increase oxidative stress (50).

The article "Adherence to lifelines diet score and risk factors of metabolic syndrome among overweight and obese adults: A cross-sectional study" was retracted in 2024. Reasons: a breach of policy by an author; concerns about the authorship.

Our study demonstrated that the consumption of fruits and vegetables was significantly higher among higher LLDS tertiles. Borgi et al. showed that higher fruit intake is associated with a lower risk of hypertension, but there was no similar link between vegetable consumption and blood pressure (54). Similarly, in a cohort study, Wang et al. demonstrated that higher consumption of fruits and vegetables was related to a decreased risk of hypertension (55). Fruits and vegetables may be linked to hypertension through a variety of mechanisms. One possible reason relates to the high flavonoid content of some fruits and vegetables (56). Macready et al. showed that a diet with high content of flavonoids from fruits and vegetables enhanced endothelium function and plasma nitric oxide while decreasing C-reactive protein and E-selectin (57). Also, fruits and vegetables high in potassium, carotenoid, vitamin C, folic acid, magnesium, and vitamin C, are thought to reduce blood pressure by enhancing endothelial function, altering baroreflex sensitivity, inducing vasodilation, and boosting antioxidant activity (58–64). Another probable explanation for this issue is that higher consumption of fruits and vegetables could influence diet composition, mainly increasing dietary fiber intake and reducing fat consumption (65).

As another finding of this study, whole grain consumption increased in higher LLDS tertiles. Whole grains may decrease the risk of high blood pressure through various mechanisms, including an enhanced insulin sensitivity and better endothelial function (66).

We also discovered that TG levels were lower in the third LLDS tertile, which included subjects with the best diet quality. Similarly, AlEssa et al. demonstrated that both DASH and alternate Mediterranean diet (aMED) patterns were linked with decreased TG contents in various quartiles (67). Several studies reported that TG, LDL-C, and blood pressure decreased with higher food quality, but HDL-C increased (68–70).

Our findings indicated no significant relationship between DBP, TC, TG, HDL-C, LDL-C, glucose, insulin, HOMA-IR, and QUICKI with LLDS. Milena et al. also reported no significant association between WC, HOMA-IR, HDL-C, and TG and diet quality evaluated by the Brazilian Healthy Eating Index (B-HEI) score (71). In contrast, Tzima et al. showed a significant decrease in TC levels in higher diet quality in an overweight/obese population (46).

The article "Adherence to lifelines diet score and risk factors of metabolic syndrome among overweight and obese adults: A cross-sectional study" was retracted in 2024. Reasons: a breach of policy by an author; concerns about the authorship.

The lack of association between LLDS as a diet quality index and metabolic indicators other than SBP was surprising in our study. The high carbohydrate content in higher tertiles of LLDS may partially explain these findings. As demonstrated in Supplementary Table 1, the percentage of total calories from carbohydrates was significantly higher in the highest tertile of LLDS. According to a cohort study (72), participants who consumed high carbohydrate diets had lower HDL-C and higher levels of TG and TC. Also, Cho and Choi (73) showed that a high carbohydrate diet was related to an elevated risk of MetS. Thus, high carbohydrate intake amongst participants in higher tertiles of LLDS may be a possible reason for the lack of association between LLDS and other metabolic risk factors other than SBP. Another possible reason can be that refined grain products were not included in the LLDS calculations and were placed in the unknown group (15). These products have a high glycemic index and glycemic load (74), and several studies have found a positive association between glycemic load and insulin resistance (75) and metabolic risk factors (76).

As far as the researchers investigated, this is the first cross-sectional study assessing the relationship between LLDS and cardiometabolic components. Nonetheless, this study had some limitations. First, due to the cross-sectional design of the study, any causal inference is difficult. Second, the study was conducted in northwestern Iran, which has particular food patterns and eating habits. So, generalizing the results to other parts of the country should be done with caution. Secondly, the difficulty and low accuracy of estimating table salt intake, when 24 urine samples were not available should also be considered in interpretation of our results. Finally, it should be noted that FFQs are ideal for long-term dietary assessment, and they are reasonable for estimating macronutrients and main micronutrients. However, they have a low sensitivity for other micronutrients.

## Conclusion

In conclusion, our results suggest that higher adherence to LLDS might be associated with lower SBP among overweight and obese adults. Thus, a higher diet quality score, determined by LLDS, can be associated with a lower risk of MetS. However, further experimental and longitudinal studies are needed to better address this associations.

## Data availability statement

The raw data supporting the conclusions of this article will be made available by the authors, without undue reservation.

The article "Adherence to lifelines diet score and risk factors of metabolic syndrome among overweight and obese adults: A cross-sectional study" was retracted in 2024. Reasons: a breach of policy by an author; concerns about the authorship.

## Ethics statement

The studies involving human participants were reviewed and approved by Ethics committee of Tabriz University of Medical Sciences. Written informed consent to participate in this study was provided by the participants’ legal guardian/next of kin.

## Author contributions

MF and AA supervised the project and were involved in manuscript revision and data collection. AA was also involved in data collection. MF and AH wrote the first draft of the manuscript and were involved in revision and data analysis. AA, RA, and MK were also involved in data collection and sample recruitment. All authors read and approved the final version of the manuscript.
